The article "Research on Video Captioning Based on Multifeature Fusion" was published in 2022. Journal: Comput Intell Neurosci.

# Research on Video Captioning Based on Multifeature Fusion

**DOI:** 10.1155/2022/1204909

**Published:** 2022-04-28

**Authors:** Hong Zhao, Lan Guo, ZhiWen Chen, HouZe Zheng

**Affiliations:** School of Computer and Communication, Lanzhou University of Technology, Lanzhou, Gansu, China

## Abstract

Aiming at the problems that the existing video captioning models pay attention to incomplete information and the generation of expression text is not accurate enough, a video captioning model that integrates image, audio, and motion optical flow is proposed. A variety of large-scale dataset pretraining models are used to extract video frame features, motion information, audio features, and video sequence features. An embedded layer structure based on self-attention mechanism is designed to embed single-mode features and learn single-mode feature parameters. Then, two schemes of joint representation and cooperative representation are used to fuse the multimodal features of the feature vectors output by the embedded layer, so that the model can pay attention to different targets in the video and their interactive relationships, which effectively improves the performance of the video captioning model. The experiment is carried out on large datasets MSR-VTT and LSMDC. Under the metrics BLEU4, METEOR, ROUGEL, and CIDEr, the MSR-VTT benchmark dataset obtained scores of 0.443, 0.327, 0.619, and 0.521, respectively. The result shows that the proposed method can effectively improve the performance of the video captioning model, and the evaluation indexes are improved compared with comparison models.

## 1. Introduction

With the rapid development of the mobile Internet and the rapid popularization of intelligent devices, from “Internet + Plus” to “AI + Plus,” the process of human informatization has entered a new stage. As a new type of user-generated content, short video has widely appeared on various social platforms. While people interact through video, some unhealthy videos such as terrorist violence and pornography take advantage of it, which seriously endanger the physical and mental health of young people. Therefore, the audit of short video content is of great significance. Most of the existing video auditing methods use manual means, but manual auditing has poor real-time performance and low efficiency. Using the deep learning for video content auditing can not only improve the accuracy of the audit but also support the video screen, text, and speech for multidimensional audit. Therefore, how to obtain the main information from short videos and convert it into natural language, analyze, and understand it has become a hot research topic in the field of text expression of video content. Video captioning is a cross-modal, cross-disciplinary research, and has been a challenging research topic in the computer and multimedia fields [1, 2]. The video captioning aims at expressing the objects, attributes, and mutual relationships presented in the video in natural language. The research has broad application prospects, including helping visually impaired people to understand visual content such as movies and short videos, and helping existing video social platforms to identify the objectionable content.

The early work of video captioning is based on the fixed template structure [3–5], which mainly includes two phases, content recognition, and sentence generation from template. The content recognition stage is to visually recognize and classify the main objects in the video. The stage of generating sentences according to the template is to match the entities identified by the content with the categories required by the template, such as subject, predicate, object, and location. However, the method relies too much on the preset template, resulting in poor flexibility in generating descriptions and the simplex sentences. Inspired by the machine translation direction encoder-decoder framework, the current mainstream methods of video captioning use convolutional neural networks (CNNs) [6–8] in advance, which are widely used in the field of object recognition and detection, to obtain visual information and generate vision representation vector, and then use recurrent neural networks (RNNs) [9–11] that have made great progress in natural language processing as the encoder to receive the visual representation vector for encoding, generate the intermediate hidden vector, and send it to the decoder composed of RNN so as to generate serialized natural language expression. For example, literature [12] uses CNN to extract the image features of each frame in the video, sends it to the RNN encoder for encoding in time sequence, generates the intermediate hidden vector, and sends it to the decoder to generate the description text of the video. Literature [13] improves the performance of the video description text network by adding explicit high-level semantic attributes of images and videos, but these attributes are extracted from a single modality, which is not enough to fully understand the video. The actual video is constructed from a number of different modal contents, which contains not only a single image information, but the information such as the motion of the object in the video, the audio in the background, and the timing of the context, and the information of different modalities. There is a high degree of correlation and complementarity between them, and these modalities cooperate with each other to provide complete information. As depicted in Figure 1(a), the example video can be described as “a person is skiing fast,” in which “fast” is highly related to sports information; in Figure 1(b), the example video can be described as “there is a train whistling out of the tunnel,” in which “whistling” is closely correlated to the audio information.

Video is a recording carrier based on static pictures, but it is a higher expression than static pictures. With the movement of the object and the camera, the composition structure and plot focus of the video screen will change accordingly, and the perspective relationship of the objects in the video will also change. This change is called the motion feature of the video; the optical flow graph of video has apparent feature invariance and contains coherent motion trajectory information. The accuracy of optical flow at the boundary and small displacement has a strong correlation to the capture of video motion information. The audio signal carried by the video is also of great significance to the video. Video dubbing can explain the main points and themes of the video in the form of sound. For example, applause and whistle can only be captured from audio information. Aiming at the problem of low accuracy of video captioning based on a single visual feature, and the high correlation and complementarity between different modal information, this article uses the fusion of multiple complementary modal information to train the video captioning model. Firstly, each frame of video in the dataset is converted into a single JPEG image, and the audio information of each extracted video is stored as an audio file in wav format. Then, the representation information of static image, audio, motion, optical flow, and other modes is extracted from the extracted modal data to cross-modal information fusion, and to generate a richer and more accurate video captioning. The main work of the research is as follows:

1. According to different video modal information, various models pretrained by large-scale datasets are used to extract static, dynamic, and audio information in video, which improves the accuracy of the text expression of the video content.
2. An embedded layer based on self-attention mechanism is designed to embed the single-mode eigenvector and learn the network parameters needed in sentence generation. The complementary information between different modes can be fitted better when encoding.
3. Two schemes of joint representation and collaborative representation are used for cross-modal feature fusion, and it is verified that the collaborative representation strategy has better experimental results in this model when fusing multiple complementary video modal information.

## 2. Related Work

The video captioning aims at analyzing, understanding, and expressing the content displayed in the video through the use of natural language. At present, the mainstream methods of video captioning are based on the “coding decoding” architecture, which can be divided into three types: methods based on visual feature mean/maximum, video sequence memory modeling, and three-dimensional convolution features.

The method based on the mean/maximum value of visual features extracts the visual features by employing the mean value or the maximum value, and then encodes the features and decodes them to generate the natural language text. Venugopalan et al. [14] adopted an LSTM-MY model that uses mean pooling to extract visual features, and its performance is improved compared with the template-based method. Dong et al. [15] proposed the ruc-uva model to solve the problem of insufficient relevance of generated text and video content. This model extracts video keywords by combining the video tagging method and then combines the keywords and video frame features as the input of the decoder, which effectively improves the accuracy of the generated text. However, these methods are difficult to capture the time-series characteristics in video clips, which could cause the loss of dynamic features easily.

The method based on video sequence memory modeling effectively solves the problem that time-series features in video clips are difficult to capture. Literature [16] adopted a temporal attention (TA) model for video data preprocessing, which combines attention mechanism in the time dimension, generates text from the resulting feature input decoder, and selects the frame with the greatest correlation with the content to be generated in a time step to make the generated sentences more adaptable. Literature [17] applies the sequence-to-sequence model to the video to text task to solve the problem of variable length of video to text, and realizes the end-to-end video description of video frame sequence input and text sequence output. Although this type of model can realize the time-series feature extraction and end-to-end training of the language module, the CNN feature could easily lead to the destruction and loss of the spatial information in the video frame after the sequence transformation.

The method based on 3D convolution features can mine the static and temporal dynamic features of video at the same time by encoding the spatiotemporal features of video. In literature [18], the proposed model uses the 3D convolutional network to extract the three-dimensional features of different video segments, calculates the average value of multiple three-dimensional feature vectors, and then combines them with the average value of the CNN feature extracted from the video frame as the feature representation of the video. The features extracted by the 3D convolution network contain some dynamic information of video, which improves the performance of the model to a certain extent. Literature [19] proposed the *M*^3^ − inv3 model that jointly models visual information and language information by extracting the 2D and 3D features of the video frame, which better solved the problem of the long-term dependence of multimodal information and semantic dislocation in LSTM. Literature [20] proposes a hierarchical LSTM with the adaptive attention method for image and video captions, which uses spatial or temporal attention to select regions to predict related words. Literature [21] presents a grammar prediction action module that combines the region target features with the spatial location information of the corresponding region to form a new region target feature to guide the description generation. To further selectively integrate semantic features into the description generation model, Ryu et al. (2021) [22] used semantic alignments to establish the correlation between a word phrase and a video frame and used semantic focusing mechanism to group semantically related frames. The visual and semantic features are then passed to the codec to generate the description.

The proposed model does not fully utilize the extracted single-mode representation information and take into account the audio information carried by the video to the model. Therefore, considering the complementarity between single-mode feature parameter learning and video multimodal representation information, the semantic attributes expressed by each mode are obtained by extracting the representation information of multiple modes of video, so as to improve the performance of the video captioning model.

## 3. Video Captioning Model

### 3.1. Model Structure

The structure of the cross-modal video captioning model based on multilayer attention is shown in Figure 2. It mainly includes four parts: video preprocessing, single-modal feature extraction, coding (single-modal information embedding, multimodal information fusion), and decoding. Among them, the video preprocessing module mainly extracts the video frame and the video audio information. The single-mode feature extraction module uses the improved ResNet network [23], FFmpeg, two-stream inflated 3D convolution network [24] (I3D) to extract 2D frame features, audio MFCC features, and optical and 3D motion features of the video after increasing channel attention. The designed embedded layer is composed of a self-attention mechanism [25] and a two-layer LSTM network [26], and the encoder takes the feature vectors of the frame, motion, and audio modes as input, feeds different modal features into the embedded layer for single-mode modeling, and finally codes them into three hidden vectors {*h*_*v*_, *h*_*I*3  *D*_, *h*_audio_} and maps the information of multiple modes together to a single multimodal vector space *V*_*multi*_ through collaborative representation. The decoder receives *V*_multi_ for decoding, predicts the hidden state of the current time, outputs the probability distribution vector of each time step in turn, and uses the greedy search algorithm to take the word with the highest probability at each time step at the decoding time as the predicted output result. The word probability model of time *T* is shown in

(1) $$\begin{array}{c} P_{t}{\left(Y\right)}_{t}=\arg\max\left(softmax\left(h_{t},Y_{t-1},V_{multi}\right)\right), \end{array}$$

where *h*_*t*_ is the current hidden state, *Y*_*t*−1_ is the result of the last time step, *V*_*multi*_ is a unified multimodal vector space, *soft*max is a normalized exponential function, mapping the result to (0,1) as a probability value, and *P*_*t*_(*Y*_*t*_) represents the probability distribution of each word in the current time step. When all probability distributions are calculated, the greedy search algorithm is used to extract the word with the highest probability in each time step at the decoding time as the prediction output until the output is 〈*eos*〉 and the decoding is completed.

### 3.2. Feature Extraction

Video data differ from picture data in that video is multiframe snapshot, which makes video more suitable for describing continuous actions or pictures. Meanwhile, the video is attached with corresponding real-time sound information, so that the video can record an event more stereoscopically and vividly. Compared to a single image, the video contains not only spatial features but also temporal features, as well as audio and motion features. Because the continuous frame structure in the video conveys a wealth of information, it is difficult to determine in the context of the more significant content to accurately describe. For this reason, we use multimodal features of video to express video content text.

For the static feature extraction of video frames, a channel attention framework unit squeeze and excitation (SE) proposed in literature [27] is added to the residual network ResNet152 network [28] to extract frame-level 2D features.

For the extraction of dual-stream 3D features of video, the two-stream inflated 3D convolution network (I3D) proposed by the DeepMind team is adopted [29]. This network structure adds the idea of dual stream into 3D convolution, which can make the network better extract the spatiotemporal information of video and capture fine-grained temporal features.

For the extraction of audio information in the video, FFmpeg is used to extract the Mel frequency cepstral coefficient (MFCC) of the voice signal.

#### 3.2.1. Channel Attention

The attention mechanism in deep learning draws lessons from the human visual system. For example, the human visual system tends to focus on the key information that assist judgment in the image and ignore the irrelevant information [30]. Therefore, the attention mechanism is essentially similar to the human selectivity mechanism. Attention in deep learning refers to the weight of learning parameters The core task is to select the information more related to the current model goal from the extracted information. The extraction of video frame-level features actually extracts different information from each frame picture in different channels, so adding channel attention can give greater weight to important features. In the SE module [27], the interdependence between channels is explicitly modeled and the channel-type feature response is adaptively recalibrated. Through this mechanism, the model can learn to use global information to selectively emphasize important features and suppress redundant features. SE module realization and its structure are shown in Figure 3.

In the SE module, there are three key operations: squeeze, excitation, and reweight. In Figure 3, (a) network input matrix *X* is given, and its characteristic channel is *C*′. After a series of convolution and other operations, a characteristic diagram with the number of characteristic channels of *C* is obtained. Then, the three operations of the SE module are used to recalibrate the previously obtained feature map *U*.

The first is the squeeze operation. This operation compresses the feature map *U* along the spatial dimension. The two-dimensional information of each characteristic channel is compressed into a real number *Z*_*C*_, which has a global receptive field to a certain extent. *Z*_*C*_ represents the global information of the response on the characteristic channel. Formally, the statistic *Z*_*C*_ is generated by reducing the space dimension (*H∗W*) of the characteristic graph *U*, so the cth element of *z* is calculated in the following:

(2) $$\begin{array}{c} Z_{C}=F_{sq}\left(U_{c}\right)=\frac{1}{H\times W}\sum_{i=1}^{H}\sum_{j=1}^{W}u_{c}\left(i,j\right). \end{array}$$

In order to take advantage of the information gathered in the squeeze operation, the second important operation exception is carried out. The exception is similar to the design of the gate in the cyclic neural network structure. This operation aims at capturing the channel dependence completely. The excitation operation is implemented with two fully connected (FC) structures to reduce the model complexity and to improve the model generalization ability. The first FC layer reduces the *C* channel into *c*/*r* channels, and the dimension reduction factor *r* is a super parameter. The second FC layer is used to restore the original dimensions of the feature map. Finally, a weight coefficient *S* is obtained, which is calculated as in the following equation:

(3) $$\begin{array}{c} S=F_{ex}\left(z,w\right)=\sigma \left(g\left(z,w\right)\right)=\sigma \left(w_{2}\delta \left.\left(w_{1}z\right)\right)\right), \end{array}$$

where *σ* represents the sigmoid function and *δ* represents the ReLU function, *w*_1_ ∈ *R*^*c*/*r*×*c*^, *w*_2_ ∈ *R*^*c*×*c*/*r*^

Finally, the reweight operation is performed. The weight output from the previous operation is weighted to the previously obtained feature map *U* channel by channel, and the recalibration of the original feature on the channel dimension of the feature map is completed to obtain the final attention feature ${\tilde{X}}_{C}$. The calculation of ${\tilde{X}}_{C}$ is shown in the following equation:

(4) $$\begin{array}{c} {\tilde{X}}_{C}=F_{scale}\left(u_{c},s_{c}\right)=s_{c}\cdot u_{c}, \end{array}$$

where *F*_scale_ refers to the channel multiplication between the attention weight *s*_*c*_ and the feature map *u*_*c*_.

The SE module finally performs an attention or gating operation in the channel dimension. This attention mechanism allows the mode to pay more attention to the channel features with the largest amount of information and suppress the unimportant channel features.

#### 3.2.2. Feature Extraction of Video Frame

For the video frame feature extraction part, the SE (squeeze and excitation) module is added to the improved ResNet152 network structure and used as the video frame feature to extract the network. As shown in Figure 4, the SE module is embedded in the ResNet152 network to readjust the important features extracted by the network, so that the global information can be used to measure the importance of each feature and obtain the correlation between two channels, so as to assist in the recalibration of features. In order to simplify the complexity of model parameters, a 1*∗*1 full connection layer is adopted at both ends of the ReLU activation function of the SE module [31]. The advantages of this approach are as follows: (1) making the network more nonlinear and better fitting the complex correlations between channels; and (2) promoting useful features and suppressing features that are of little use to the current task.

Each video in the dataset is preprocessed into fixed frames, and 80 of them are taken as sample frames at equal intervals. Then, these sample frames are sent to the SE-ResNet model pretrained on the large-scale image dataset ImageNet to extract the feature information of the frames and obtain a high-dimensional feature vector of 80*∗*2048.

#### 3.2.3. Feature Extraction of Two-Stream I3D

Two-stream inflating 3D convolution network [29] I3D is one of the latest 3D convolutional networks proposed by the deep mind team. Since two-stream can capture action information simply and effectively, this network structure adds the idea of dual stream to construct an I3D network in 3D convolution. One 3D structure is used to receive RGB information, and the other is used to receive optimized smooth optical flow information. These two 3D convolution structures are derived by improving the 2D convolution structure Inception v1, as shown in Figure 5(a). The convolution kernel parameters in the 2D structure are repeated in the time dimension to form the parameters of the 3D convolution kernel, and then, the parameters are divided by *N* to ensure that the network output is the same as the 2D convolution. Therefore, the convolution kernel and pooling increase the time dimension, and other nonlinear layer structures remain unchanged. The network connection details are shown in Figure 5(b). Although 3D convolution can learn the time features of a video directly, it only performs pure forward propagation, and the optical flow algorithm provides some iterative ideas in it, the recognition accuracy of the network can be improved by adding optical flow.

Each video in the dataset is preprocessed into a 224*∗*224 fixed frame and sent it to the I3D model pretrained on the large-scale image dataset ImageNet and the video dataset kinetics to extract the dynamic features of the video to obtain a feature vector.

#### 3.2.4. Feature Extraction of Audio MFCC

At present, the commonly used speech feature extraction methods include linear prediction cepstral coefficient extraction method [32], linear predictive cepstral coefficient (LPCC), and Mel frequency cepstral coefficient extraction method [33], and Mel frequency cepstral coefficient (MFCC). MFCC was proposed by Stevens, Volkman, and Newman in 1937. MFCC is mainly based on human nonlinear auditory mechanism to simulate the function of the human ear for speech frequency analysis, so as to better extract speech signal features. Mel is the measurement unit of perceived tone or tone frequency, and 1 Mel is 1/1000 of the tone perception degree of 1000 Hz. The specific definition is shown in the following equation:

(5) $$\begin{array}{c} f_{mel}=2595\log_{10}\left(1+\frac{f_{Hz}}{700}\right),\\ f_{mel}=1125\;\ln\left(1+\frac{f_{Hz}}{700}\right), \end{array}$$

where *f*_*Hz*_ is the actual linear frequency and *f*_mel_ is the Mel frequency standard.

The cepstrum parameter feature of the Mel filter plays an important role in speech feature extraction. Its calculation is simple, and its discrimination ability is prominent. The feature parameter extraction principle of MFCC is shown in Figure 6.

First, the audio signal extracted from the dataset is preprocessed, such as pre-emphasis, framing, and windowing, and then, the corresponding discrete Fourier transform is performed on the single frame signal after framing to obtain the frequency-domain data, as shown in the following equation:

(6) $$\begin{array}{c} X_{\text{i}}\left(k\right)=\sum_{n=1}^{N}x_{i}\left(n\right){\mathrm{\&ExponentialE;}}^{\frac{-j^{2}\pi nk}{N}};1\leq k,n\leq N, \end{array}$$

where *x*(*k*) represents the time domain signal; *x*_*i*_(*k*) is the data of the *i-*th frame; and *K* represents the *k*th spectral line in the frequency domain.

Secondly, the frequency-domain data obtained above are filtered by *W* Mel frequency filters, and the spectrum, Mel filter banks, and frequency envelope are extracted. The frequency-domain response of the filter *H*_*w*_(*k*) is in the following equation:

(7) $$\begin{array}{c} H_{w}\left(k\right)=\left\{\begin{array}{cc} 0, & k<f\left(w-1\right)\\ \frac{2\left(k-f\left(w-1\right)\right)}{\left(f\left(w+1\right)-f\left(w-1\right)\right)\left(f\left(w\right)-f\left(w-1\right)\right)}, & f\left(w-1\right)\leq k<f\left(w\right)\\ \frac{2\left(f\left(w+1\right)-k\right)}{\left(f\left(w+1\right)-f\left(w-1\right)\right)\left(f\left(w\right)-f\left(w-1\right)\right)}, & f\left(w\right)\leq k\leq f\left(w+1\right)\\ 0, & k>f\left(w+1\right) \end{array}\right., \end{array}$$

where ∑*H*_*W*_(k)=1; *f*(*w*) is the center frequency of the filter.

Then, the logarithm of the processed energy spectrum is taken so that the amplitude multiplication in the Fourier transform is converted into addition to obtain the logarithmic energy, which is calculated in the following equation:

(8) $$\begin{array}{c} S_{i}\left(w\right)=\ln\left(\sum_{k=0}^{N-1}{\left|X_{i}\left(k\right)\right|}^{2}H_{w}\left(k\right)\right);0\leq w<W, \end{array}$$

where *i* is the *i*-th frame and *k* is the *k-th* spectral line in the frequency domain.

Finally, it is substituted into the discrete cosine transform (DCT) to obtain the MFCC coefficient, which is calculated in the following equation:

(9) $$\begin{array}{c} MFCC\left(i,n\right)=\sum_{w=0}^{W-1}S\left(w\right)\cos\left(\frac{\pi n\left(w+0.5\right)}{W}\right),0\leq w<W,n=1,2,\ldots \ldots ,L. \end{array}$$

where *W* is the *w*-th Mel filter, *i* is the *i*-th frame, and *n* is the spectral line obtained after DCT.

The audio extracted from each video in the dataset is divided into 1120 frames, and the MFCC signal of 20 dimensions is extracted from each frame and stored as an 1120*∗*20 high-dimensional audio feature matrix.

### 3.3. Feature Fusion

The information fusion of different modes is a key point in multimodal research, which integrates the information extracted from different modes into a stable multimodal representation. There are two multimodal feature fusion strategies [34]: joint representations and coordinated representations.

Joint representation is shown in Figure 7; this method maps the information of multiple modes together into a unified multimodal vector space. After multiple modal features *x*_1_, ....., *x*_*m*_ are obtained, the characteristic *X*=*f*(*x*_1_, ....., *x*_*m*_) is obtained by splicing and fusing. When the splicing vector dimension is high, principal component analysis (PCA) dimensionality reduction operation is carried out to form a multidimensional feature vector space *F*=*PCA*(*X*).

Collaborative representation is shown in Figure 8. Instead of seeking fusion, this method models the correlation among various modal data but maps the information of multiple modalities to a collaborative space, which is expressed as *f*(*x*_1_) ~ *f*(*x*_*n*_), where ∼ represents a collaborative relationship. The goal of network optimization is to optimize the cooperative relationship.

As shown in Figure 2, the various modal features extracted from the pretraining model are input into the embedded layer based on the self-attention mechanism for single-mode parameter learning. Then, the extracted multimodal feature vectors are fused by the above two fusion methods. As shown in Table 1, in the ablation experiment results, it is found that for the field of video captioning, the performance of cooperative representation and fusion of multimodal features is better than joint representation. The joint representation structure retains the independent representation space of multiple modes, which is more suitable for applications with only one mode as input, such as cross-modal retrieval and translation. However, the cooperative representation structure pays more attention to capture the complementarity of multimodes and obtains multimode representation *X* by fusing multiple input modes *X*, which is more suitable for multimode as input.

## 4. Experimental Design and Result Analysis

### 4.1. Experimental Hardware Platform

In this experiment, the server CPU is 48-core Intel(R) Xeon(R) Gold 5118, the running memory is 128G, the GPU card is NVIDIA Tesla V100, the video memory is 32G, and the operating system is Ubuntu18.04. NVIDIA CUDA 11.3, cuDNN V8.2.1 deep learning acceleration library, and PyTorch deep learning framework supporting GPU acceleration are installed.

### 4.2. Datasets

#### 4.2.1. MSR-VTT

MSR-VTT [35] is a large public dataset released by Microsoft in 2016 for research into video-generated text. We used the updated MSR-VTT from the 2017 competition, which contains 10,000 training video clips and 3,000 test video clips for a total of 41.2 hours. On average, each clip contains 20 natural language tags, 200000 statements in total. The dataset contains the most comprehensive and representative video content that consists of 257 popular categories from 20 representative categories (including cooking and movies) of the real video search engine, which is conducive to enhance and verify the generalization ability of the video semantic description algorithm. The content distribution of the dataset is shown in Figure 9. The *x*-axis is the video category, a total of 20 categories, and the *y*-axis is the total number of videos under each category.

#### 4.2.2. Large-Scale Movie Deion and Understanding Challenge Dataset

The large-scale movie description challenge LSMDC dataset is based on the joint presentation of MPII Movie Description Dataset (MPII-MD) [36] and Montreal Video Annotation Dataset (M-VAD) [37]. The dataset contains more than 128K sentence fragment pairs and 158-h video. The training, validation, public, and blind test sets contain 101079, 7408, 10053, and 9578 video clips, respectively. Since the vocabulary used to describe action movies may be quite different from those used in comedy movies, this division balances the types of movies in each group, making the data more evenly distributed.

### 4.3. Evaluation Metrics

For model performance evaluation, four algorithms widely used in the field of video caption, namely, consensus-based image description evaluation (CIDEr) [38], Metric for Evaluation of Translation with Explicit Ordering (METEOR) [39], Recall-Oriented Understudy for Gisting Evaluation Longest Common Subsequence (ROUGEL) [40], and Bilingual Evaluation Understudy (BLEU) [41], are used as evaluation indicators to calculate evaluation scores for the model in this article and the comparison model, thereby objectively evaluating the effect of the model's sentence description generation.

### 4.4. Experimental Parameters and Result Analysis

#### 4.4.1. Experimental Parameter Settings

Scaling the extracted original frame size to 256*∗*256 pixels before the model reads each frame. When extracting features, perform 15° random rotation on each frame of the image, which is needed firstly, and then perform random clipping to obtain an image with the size of 224*∗*224 pixels. Summarize and count the text vocabulary after the word segmentation, and then form a vocabulary list that consists of the words that are larger than the low-frequency threshold, and remove the vocabulary below the low-frequency threshold. Finally, select the vocabulary threshold as 5 and get 16860 words.

In the training phase of the model, Adam's algorithm [42] is used to optimize the parameters of the model. The parameters of the optimizer are *α*=0.9, *β*=0.999, *ε*=10^−8^. The initial learning rate of the model is 0.001, and the learning rate decay rate is 0.8. The model is trained with a learning rate decay of 0.8 for 50 consecutive rounds without loss, and the negative log-likelihood loss function is used to measure the distance between the labeled statements of the dataset and the generated statements of the model, and the batch size is set to 128. The single-mode embedding layer adopts a two-layer LSTM network, and the numbers of LSTM layers of the fusion feature encoder and decoder are set to 1, 2, and 3.

#### 4.4.2. Analysis of Experimental Results

During the training of the model, the average loss value is kept every 50 rounds. The curve of the loss value is shown in Figure 10. The initial loss decreases obviously. After 2300 rounds of training, the overall loss value tends to be stable.

To verify the validity of the model and the impact of specific parameters on the model, two-mode *V*_*f*_+*V*_*I*3  *D*_, *V*_*f*_+*V*_audio_ and three-mode *V*_*f*_+*V*_*I*3  *D*_+*V*_audio_ video captioning models were trained for static frame feature *V*_*f*_, motion feature *V*_*I*3  *D*_, and MFCC feature *V*_audio_ of the video. On the basis of each mode combination, the number of layers of LSTM network is set as 1 layer, 2 layers, and 3 layers for the single-mode embedded module and encoder module, and the model training experiments are carried out, respectively. The model comparison experiment is carried out under the MSR-VTT dataset, and the experimental results are shown in Table 1. Through nine sets of experiments, it can be seen that the monomodal embedding-multimodal fusion video captioning model constructed in this study can optimize the model by learning the parameters of monomodal information and fusing the representation information of multiple complementary modalities. The performance of the model also proves that there is a high degree of correlation and complementarity among different modal information. According to the data in the table, when the number of LSTM layers is fixed, the fusion of three complementary modal information including 2D frame features, I3D features containing 3D and optical flow information, and MFCC features of audio have the highest evaluation score for the model. When the mode is fixed, selecting 2 layers of LSTM layers in the embedded layer and encoder module is the best for the experiment. In the case of fixed modes and the number of layers of the LSTM network, the model trained by cooperative representation has a higher test score than that obtained by joint representation, which proves that the effect of modal information fusion by cooperative representation in the video captioning is better. The experimental results show that the joint representation structure retains independent representation space of multiple modes and is more suitable for applications with only one mode as input, such as cross-modal retrieval and translation. The cooperative representation structure pays more attention to capture the multimode complementarity, fusing multiple input modes *x*_1_, ....., *x*_*m*_ to obtain the multimode representation *X*=*f*(*x*_1_, ....., *x*_*m*_), which is more suitable for multimode as input.

First, three modal features are fed into the embedded layer structure to learn the parameters that related to the single mode. Then, the multimodal information is fused through the joint representation and fed into the encoder-decoder. The ablation results show that the performance of the model is improved by fused audio information compared with single-mode and dual-mode cases. Compared with the single-mode fusion score evaluation indexes BLEU4, METEOR, ROUGEL, and CIDEr increased by 0.137, 0.072, 0.102, and 0.130, respectively. Compared with dual-mode fused score evaluation index, BLEU4, METEOR, ROUGEL, and CIDEr are improved by 0.084, 0.113, 0.016, and 0.124, respectively.

This study is compared with the top five model structures in the second MSR-VTT challenge, and the results are shown in Table 2.

This article also compares the results with the representative research work in the field of video captioning, as shown in Table 3.

As can be seen from Tables 2 and 3, in the evaluation indexes such as BLEU4, METEOR, ROUGEL, and CIDEr, the model improved 0.139, 0.114, 0.125, 0.315, respectively, compared with the top five models in the MSR-VTT challenge. Compared to the authoritative models in this field, the proposed model improves 0.158, 0.090, 0.099, and 0.171, which verifies the performance improvement of the video captioning model and the superiority of the proposed model.

This article also conducts experiments based on the latest large-scale movie description challenge (LSMDC) dataset.  Table 4 shows the comparison of the METEOR results of the model on the LSMDC public dataset.

The model extracts multiple modal information of the video and uses it to train the model so that the model can obtain more complementary and diversified characterization information, making the model more robust and adaptable to multiple types of video clips. The text description is more specific and accurate, which further proves that the different modal information of the video has a high degree of correlation and complementarity.

In the split test set from the MSR-VTT dataset, different categories of video were selected.  Figure 11 shows the effect of the text generation of the video content under four different categories, and each dataset selected the first five true markup statements (ground truth, GT), from which the visual model is generated to improve the accuracy and richness of video content text generation, and it shows that the performance of the model is improved by the fusion of multiple complementary modes.

## 5. Conclusion

In this article, a single-mode embedding multimode fusion video captioning model is proposed. Through a variety of efficient pretraining models, various modal representations contained in the video are effectively extracted, and static frame information, dynamic 3D, optical flow information, and audio information are complementary. The embedded layer based on self-attention is designed to learn the characteristic parameters of a single mode, which can enhance the complementarity of each mode better. Provide comprehensive and plentiful representation information for video generation text. And make the model generate more rich and accurate natural language. The above methods are verified by a series of ablation experiments and comparative experiments on MSR-VTT and LSMDC datasets. The experimental results show that the performance of the proposed model is significantly better than other models, and the generated text is more accurate.

In the later research work, we will make further improvements on the method of cross-modal information fusion and the complementarity of modal information. Combined with the attention mechanism to do further improvement work, make the alignment of various modal information with the text more accurate, and make the model obtain more accurate and rich representation information, so as to generate high-quality text and ensure the lightweight of the model.

## Figures and Tables

**Figure 1:** The video contains not only physical objects, but also features such as sound. When we pay more attention to these supplementary features, the generated text will be more complete. (a) Video example of fast skiing. (b) Video example of a train honking out of a tunnel.

**Figure 2:** The architecture of the MM-V2T (multimodal video content text generation model). Specifically, the MM-V2T is composed of three parts as follows: video preprocessing, single-modal feature extraction, coding (single-modal information embedding, multimodal information fusion), and decoding.

**Figure 3:** SE network structure.

**Figure 4:** ResNet original structure and ResNet structure embedded with SE module.

**Figure 5:** Three-dimensional convolution and two-stream expansion 3D convolution network structure. (a) 3D Incception V1. (b) I3D.

**Figure 6:** MFCC feature parameter extraction.

**Figure 7:** Joint representation.

**Figure 8:** Collaboration representation.

**Figure 9:** MSR-VTT dataset content distribution.

**Figure 10:** Decline curve of the training loss value.

**Figure 11:** Dataset test visualization case.

**Table 1:** Comparison of the experimental results of the model obtained by different experimental parameters and different modal information fusion training under the MSR-VTT dataset.

Number layer	Feature	Score							
		BLEU4		METEOR		ROUGEL		CIDEr	
		Coordinated	Joint	Coordinated	Joint	Coordinated	Joint	Coordinated	Joint
1	*V*_*f*_+*V*_*I*3 *D*_	0.306	0.299	0.255	0.251	0.517	0.518	0.391	0.400
	*V*_*f*_+*V*_*au* *di* *o*_	0.359	0.352	0.214	0.200	0.603	0.598	0.397	0.395
	*V*_*f*_+*V*_*au* *di* *o*_+*V*_*I*3 *D*_	0.401	0.410	0.290	0.287	**0.619**	0.586	0.422	0.410

2	*V*_*f*_+*V*_*I*3 *D*_	0.334	0.325	0.235	0.220	0.520	0.499	0.394	0.396
	*V*_*f*_+*V*_*au* *di* *o*_	0.386	0.381	0.243	0.244	0.609	0.587	0.424	0.422
	*V*_*f*_+*V*_*au* *di* *o*_+*V*_*I*3 *D*_	**0.443**	0.430	**0.327**	0.319	0.612	0.600	**0.521**	0.517

3	*V*_*f*_+*V*_*I*3 *D*_	0.325	0.319	0.227	0.231	0.542	0.539	0.389	0.391
	*V*_*f*_+*V*_*au* *di* *o*_	0.379	0.377	0.246	0.237	0.597	0.585	0.463	0.459
	*V*_*f*_+*V*_*au* *di* *o*_+*V*_*I*3 *D*_	0.393	0.390	0.292	0.293	0.599	0.571	0.497	0.469

**Table 2:** Comparing the experimental results with the top five model structures in the second MSR-VTT challenge.

Rank	Organization	BLEU4	METEOR	ROUGEL	CIDEr
1	RUC&CMU	0.390	0.255	0.542	0.315
2	TJU	0.359	0.226	0.515	0.249
3	NII	0.359	0.234	0.514	0.231
4	Tongji University	0.351	0.226	0.509	0.236
5	IIT Delhi	0.304	0.213	0.494	0.206
	**Ours**	**0.443**	**0.327**	**0.619**	**0.521**

**Table 3:** Comparing the experimental results with the representative research work in the field of video captioning.

Models	BLEU4	METEOR	ROUGEL	CIDEr
MPool [14]	0.304	0.237	0.520	0.350
Ruc-uva [13]	0.387	0.269	—	0.459
S2VT [17]	0.314	0.257	0.559	0.352
TA [16]	0.285	0.250	0.533	0.371
SAAT [21]	0.399	0.277	0.612	0.510
M^3^-Inv3 [19]	0.381	0.266	—	—
SGN [22]	0.408	0.283	0.608	0.495
PickNet [12]	0.389	0.272	0.595	0.421
**Ours**	**0.443**	**0.327**	**0.619**	**0.521**

**Table 4:** In this article, the model is compared with the experimental results of the large-scale film description challenge in the LSDC dataset.

User or model	Meteor
frcnnBigger	0.033
rakshithShetty	0.046
EITanque	0.056
Yj	0.070
S2VT	0.070
**Ours**	**0.072**

## Data Availability

The experimental data used to support the findings of this study are available from the corresponding author upon request.
